This article has been retracted.

# Ultrasound Multiparametric Assessment of the Impact of Hypertensive Disorders of Pregnancy on Fetal Cardiac Function and Growth and Development

**DOI:** 10.1155/2022/3419966

**Published:** 2022-06-06

**Authors:** Maoting Lv, Shanshan Yu, Yongzhen Li, Xiaoting Zhang, Dan Zhao

**Affiliations:** ^1^Second Department of Ultrasound Diagnosis, Cangzhou Central Hospital, Cangzhou, China; ^2^Delivery Room, Cangzhou Central Hospital, Cangzhou, China; ^3^Second Department of Neurosurgery, Cangzhou Central Hospital, Cangzhou, China

## Abstract

**Objective:**

To evaluate the ultrasound multiparametric assessment of the impact of hypertensive disorders of pregnancy (HDP) on fetal cardiac function and growth and development.

**Methods:**

In this prospective study, 98 cases of HDP treated in our institution were recruited into a study group, and 100 pregnant women with healthy singleton pregnancies were included in a control group. All eligible patients were also assigned to either study group A (HDP fetuses with growth restriction) or study group B (HDP fetuses with normal growth). Fetal echocardiography was performed on all eligible participants to obtain hemodynamic and cardiac function parameters for the evaluation of fetal growth and development, and the impact of HDP on fetal heart function and growth and development was analyzed.

**Results:**

HDP fetuses were associated with smaller head circumference, biparietal diameter, femoral length, and abdominal circumference versus healthy fetuses. The study group had a higher resistance index (RI) and pulsatility index (PI) of umbilical artery (UA), ductus venous (DV), pulmonary vein (PV), and lower RI and PI of aortic isthmus (AoI) than the control group. The study group showed higher left and right ventricular isovolumic contraction time (IVCT), isovolumic relaxation time (IVRT), and myocardial performance index (MPI) values and lower mitral and tricuspid *E* wave and *E*/*A* values than the control group. The systolic blood pressure was positively correlated with PI, RI of UA, DV, and PV, and left and right ventricular IVCT, IVRT, and MPI and negatively correlated with PI and RI of AoI and mitral and tricuspid *E* wave and *E*/*A* values of HDP fetuses. The peak systolic/diastolic flow rate (S/D), PI, and RI of umbilical blood flow in study group A were higher than those in study group B. Umbilical blood flow *S*/*D* showed the highest AUC and specificity for predicting fetal growth restriction, and PI had the highest sensitivity for predicting fetal growth restriction.

**Conclusion:**

HDP compromises fetal cardiac function and growth, and ultrasound multiparametric assessment provides accurate detection of fetal cardiac function and hemodynamics changes. The patient's condition can be monitored through the assessment of ultrasound parameters of fetal growth and development.

## 1. Introduction

Hypertensive disorder of pregnancy (HDP) is a common comorbidity during pregnancy, with hypertension, proteinuria, and edema as the main clinical manifestations [1] and is an obstetric complication unique to pregnant women, resulting in a serious threat to maternal and fetal health and life. It is also an important cause of adverse birth outcomes such as preterm delivery, low birth weight, and perinatal mortality [2, 3]. HDP presents multifactorial pathogenesis with various maternal underlying pathological conditions and is susceptible to environmental factors during pregnancy [4]. The 2018 guidelines for the classification, diagnosis, and management of HDP issued by the International Society for the Study of Hypertension in Pregnancy classify HDP as hypertension in pregnancy and preeclampsia [5]. HDP contributes to maternal cardiac damage and predisposes to impaired placental circulation and symptoms of ischemia and hypoxia [6], leading to abnormal fetal cardiac function and fetal growth restriction [7, 8]. Medical ultrasonography is an ultrasound-based diagnostic medical imaging technique that enables the visualization of muscles and internal organs, including their size, structure, and pathological lesions [9, 10]. Ultrasound is a commonly used obstetric test to identify structural and functional abnormalities of the fetal heart and facilitates the assessment of the effects of HDP on fetal cardiac function [11, 12]. This study was to evaluate the ultrasound multiparametric assessment of the impact of HDP on fetal cardiac function and growth and development.

## 2. Materials and Methods

### 2.1. Baseline Data

In this prospective study, 98 cases of HDP treated in our institution between May 2019 and June 2020 were recruited into a study group, and 100 pregnant women with healthy singleton pregnancies were included in a control group. All eligible patients were also assigned to either study group A (HDP fetuses with growth restriction) or study group B (HDP fetuses with normal growth). The baseline characteristics of the study group (aged 24–35 years, mean age of 28.17 ± 4.02 years, gestational weeks of 26–30 weeks, mean gestational weeks of 28.01 ± 1.81 weeks) were comparable with those of the control group (aged 24–34 years, mean age of 28.05 ± 4.18 years, gestational weeks of 26–30 weeks, mean gestational weeks of 28.15 ± 1.41 weeks) (*P* > 0.05) (Table 1). This study was approved by the Ethics Committee of the Cangzhou Central Hospital, No. 2019-13-179.

### 2.2. Inclusion and Exclusion Criteria

Patients who met the diagnostic criteria of HDP formulated by the International Society for the Study of Hypertension in Pregnancy in 2018; patients with singleton pregnancies; and patients who provided written informed consent were included.

Subjects with incomplete clinical data; subjects with diabetes mellitus and nephritis; and subjects with inborn mental retardation or mental illness were excluded.

### 2.3. Methods

The examination apparatus was a color Doppler ultrasound diagnostic instrument (GE, USA) with a 3D volumetric probe frequency of 4–8 MHz. The subject laid flat on her back to expose her abdomen and maintained stable breathing. Two-dimensional gray-scale ultrasound scanning was performed to measure fetal head circumference, biparietal diameter, femoral length, and abdominal circumference and to calculate gestational age. The tissue multispectral imaging mode was activated and the sampling volume was adjusted to the appropriate width to measure the resistance index (RI) and pulsatility index (PI) of the umbilical artery (UA), aortic isthmus (AoI), ductus venous (DV), and pulmonary vein (PV), isovolumic contraction time (IVCT), isovolumic relaxation time (IVRT), and ejection time (ET) of the fetal left and right ventricles. The fetal mitral and tricuspid peak filling maximum filling velocity in early diastole (*E* wave) and late diastolic peak maximum filling velocity (*A* wave) were also obtained, and the right ventricular myocardial performance index (MPI) and the *E*/*A* value were calculated. An umbilical artery flow test was performed at 28–36 weeks of gestation. The subject emptied the bladder and laid flat on the back with the abdomen exposed. The fetal position was checked and the probe was placed on the abdomen for examination, and the umbilical artery flow sonogram was probed on the ventral side of the fetus. When a typical and stable waveform appeared, the waveform was frozen. More than 5 peaks and valleys of the same spectrogram were selected to record the umbilical blood flow *S*/*D*, and the average value was obtained for 3 consecutive measurements.

### 2.4. Statistical Analysis

SPSS22.0 software was used for data analyses. The count data are expressed as (n (%)) and analyzed using the chi-square test. The measurement data are expressed as (*x* ± *s*) and analyzed using Students' *t*-test. The Pearson method was used for correlation analysis. The differences were considered statistically significant at *P* < 0.05.

## 3. Results

### 3.1. Clinical Data

The systolic blood pressure, diastolic blood pressure, and 24 h urine protein quantification of the study group (152.65 ± 7.16, 101.47 ± 4.28, 3.08 ± 0.77) were higher than those in the control group (108.34 ± 6.12, 62.37 ± 4.53, 0.08 ± 0.02) (*P* < 0.05) (Table 2).

### 3.2. Fetal Growth and Development

The HDP fetuses were associated with smaller head circumference, biparietal diameter, femoral length, and abdominal circumference (31.65 ± 2.81, 8.82 ± 0.76, 6.79 ± 0.58, 30.88 ± 3.29) versus healthy fetuses (32.94 ± 1.93, 9.18 ± 0.53, 7.02 ± 0.53, 32.77 ± 2.38) (*P* < 0.05). (Table 3).

### 3.3. Ultrasound Hemodynamic Parameters

The study group had higher RI and PI of UA, DV, and PV, lower RI and PI of AoI (0.89 ± 0.18, 0.63 ± 0.17, 0.68 ± 0.11/1.21 ± 0.23, 0.86 ± 0.19, 1.03 ± 0.18, and 0.71 ± 0.10/1.96 ± 0.25) than the control group (0.66 ± 0.12, 0.48 ± 0.12, 0.52 ± 0.08/1.08 ± 0.13, 0.64 ± 0.13, 0.83 ± 0.12, and 0.87 ± 0.17/2.32 ± 0.38) (*P* < 0.05) (Table 4).

### 3.4. Fetal Heart Function

#### 3.4.1. Fetal Heart Function Parameters

The study group showed higher left and right ventricular IVCT, IVRT, and MPI values (48.33 ± 6.98, 48.86 ± 7.02, 0.53 ± 0.11/52.88 ± 12.08, 49.98 ± 11.02, 0.57 ± 0.11) and lower mitral and tricuspid *E* wave and *E*/*A* values (0.34 ± 0.09, 0.58 ± 0.11/0.32 ± 0.04, 0.51 ± 0.05) than the control group (38.65 ± 5.18, 40.91 ± 6.77, 0.42 ± 0.07/42.61 ± 9.52, 40.32 ± 8.13, 0.47 ± 0.09 and 0.34 ± 0.09, 0.58 ± 0.11/0.41 ± 0.11, 0.62 ± 0.14) (*P* < 0.05). (Table 5).

#### 3.4.2. Correlation

The systolic blood pressure was positively correlated with PI, RI of UA, DV, and PV, and left and right ventricular IVCT, IVRT, and MPI and negatively correlated with PI and RI of AoI and mitral and tricuspid *E* wave and *E*/*A* values of HDP fetuses (Table 6).

### 3.5. Fetal Growth Restriction

#### 3.5.1. Umbilical Artery Flow Parameters

The peak systolic/diastolic flow rate, PI, and RI of umbilical blood flow in study group A (3.89 ± 0.98, 1.29 ± 0.33, and 0.79 ± 0.16) were higher than those in study group B (2.50 ± 0.66, 0.91 ± 0.31, and 0.63 ± 0.08). (Table 7).

#### 3.5.2. Predictive Value

Umbilical blood flow S/D showed the highest AUC and specificity for predicting fetal growth restriction, and PI had the highest sensitivity for predicting fetal growth restriction (Table 8).

## 4. Discussion

Hypertensive disorder of pregnancy is a common comorbidity during pregnancy and is characterized by hypertension, proteinuria, and edema, which may be associated with adverse birth outcomes such as preterm delivery, low birth weight, and perinatal death [4, 13]. The pathogenesis of HDP is multifactorial, and HDP may lead to maternal cardiac damage, placental circulation disorders, systemic small artery spasm, and increased vascular permeability. Plasma exudation causes hypercoagulation of blood and atherosclerosis of blood vessels at the myometrium, which seriously compromises fetal development [5]. Systemic small vessel spasms can cause increased peripheral circulatory resistance, resulting in insufficient intrauterine blood and oxygen supply and increased left ventricular afterload, thereby inducing irreversible left ventricular hypertrophy. To protect the blood supply to vital organs of the fetus, the organism compensates for vasodilatation and enhances venous blood return, which subsequently leads to increased cardiac load [14], both of which are associated with decreased cardiac systolic function and impaired diastolic function, seriously compromising the fetal cardiac development [7, 15]. Ultrasound is a commonly used obstetric test that identifies structural and functional abnormalities of the fetal heart and helps to assess fetal cardiac function [16]. It can reflect umbilical hemodynamic correlation and fetal-placental circulatory resistance characteristics [17], which provides objective indicators of intrauterine fetal development and facilitates the identification of intrauterine fetal abnormalities [18, 19].

In the present study, HAP fetuses showed higher RI and PI of UA, DV, PV, and lower RI and PI of AoI than healthy fetuses. The results of the study by He Ying et al. indicate that HDP leads to inadequate fetal blood supply and a compensatory increase in venous blood return, resulting in increased PI and RI, and the detection of PI and RI of UA, AoI, DV, and PV in HDP patients contributed to a better understanding of fetal cardiac function, which is consistent with the results of the present study. HDP is associated with insufficient trophoblast invasion and reduced placental vascular density. To protect the brain and heart vital organs, the fetus's body dilates the brain and heart vessels through neurohumoral regulatory mechanisms to ensure blood oxygen supply, and the AoI is a critical part of fetal blood circulation, with the dual effects of cardiac contraction and peripheral circulatory resistance, so the AoI vascular bed resistance declined in the study group. The study group had higher left and right ventricular IVCT, IVRT, and MPI parameters, and lower values of mitral and tricuspid *E* and E/A parameters than the control group (*P* < 0.05), indicating more severely impaired fetal cardiac function in HDP fetuses. The development of HDP is related to intrauterine ischemia and hypoxia in the fetus, and compensatory vasodilatation increases venous blood return to protect fetal blood supply to vital organs, which increases fetal cardiac afterload [20], thereby leading to an increase in A wave and a decrease in E/A ratio. MPI provides a sensitive reflection of cardiac systolic and diastolic function, and Liu et al. found that MPI was significantly higher in late HDP fetuses versus healthy pregnant women. The results of the correlation analysis in the present study suggested that the increase in systolic blood pressure magnifies the effect of HDP on fetal cardiac function, resulting in a more severe impairment of cardiac function. Furthermore, HDP resulted in inferior fetal growth and development versus healthy fetuses. The placenta in a normal pregnancy state matures with increasing gestational weeks, in which the placental vascular resistance and umbilical blood flow *S*/*D* are decreased and the blood flow is increased to ensure the blood supply for fetal development. However, HDP leads to alterations in the placental vascular structure, with a decrease in the number of small arteries, atherosclerosis, and deposition of fibrous material, which reduces fetal-placental blood circulation, impedes intrauterine fetal development, and increases the resistance load, resulting in a significant increase in umbilical blood flow *S*/*D*. Here, umbilical blood flow *S*/*D* had the highest AUC and specificity for predicting fetal growth restriction, and PI had the highest sensitivity for predicting fetal growth restriction. Previous studies have demonstrated that assessment of fetal growth and development ultrasound parameters contribute to evaluating patients' conditions, which is consistent with the results of the present study.

The normal development of the fetus during pregnancy is closely related to the placental structure, the differentiation of cytotrophoblasts, and the normal formation of the uteroplacental vasculature. In normal pregnancy, the placenta of the uterus is vasodilated within the meconium layer and superficial muscular layer, with infiltration of cellular trophoblasts visible in the vessel wall. In contrast, patients with hypertensive disorders during pregnancy have thickened blood vessel walls and narrowed lumen in the placental bed, and infiltration of trophoblast cells into blood vessels is rarely seen. In addition, the more severe the condition of patients with severe preeclampsia, the more obvious the pathological changes in small spiral arteries. Research has found that baicalin has a therapeutic effect on gestational hypertension. Modern pharmacological studies have shown that the Chinese medicinal herb Scutellariae Radix has various pharmacological effects such as antibacterial, anti-infective, anti-inflammatory, antioxidant, sedative, and cardiovascular and endothelial damage protection. Baicalin is one of the main active ingredients of Scutellariae Radix. It was found [1] that the anti-inflammatory effect of baicalin is achieved by inhibiting the phosphorylation level of the MAPK signaling pathway and increasing the expression level of anti-inflammatory factors. Pregnant women with preeclampsia had serum-stimulated activation of p38 MAPK and JNK pathways and increased expression of endothelial cell surface adhesion molecules in human umbilical vein endothelial cells, and this activation was associated with the severity of preeclampsia. The expression of p38, JNK, and ICAM-1 increased with the aggravation of the disease. Baicalin can significantly inhibit the expression of ICAM-1 which has an injurious effect on endothelial cells in the endothelial cell injury model, which is most probably related to the inhibition of the activation of JNK and P38MAPK pathways in the MAPK signaling pathway. Thus, Scutellariae Radix was associated with a unique protective effect on endothelial cell injury.

## 5. Conclusion

HDP compromises fetal cardiac function and growth, and ultrasound multiparametric assessment provides accurate detection of fetal cardiac function and hemodynamics changes. The patient's condition can be monitored through the assessment of ultrasound parameters of fetal growth and development. The limitations of this study lie in the absence of long-term follow-up observations of fetal growth and development to obtain more data on growth and development, which will be explored in future studies.

## Figures and Tables

**Table 1:** Comparison of baseline characteristics ($\bar{x}$ ± *s*).

Groups	*N*	Age	Mean age	Gestational week	Mean gestational week
Study group	98	24–35	28.17 ± 4.02	26–30	28.01 ± 1.81
Control group	100	24–34	28.05 ± 4.18	26–30	28.15 ± 1.41
*t*	—	—	0.206	—	0.608
*P*value	—	—	0.837	—	0.544

**Table 2:** Comparison of clinical data ($\bar{x}$ ± *s*).

Groups	*n*	Systolic blood pressure (mmHg)	Diastolic blood pressure (mmHg)	24 h urine protein quantification (g/24 h)
Study group	98	152.65 ± 7.16	101.47 ± 4.28	3.08 ± 0.77
Control group	100	108.34 ± 6.12	62.37 ± 4.53	0.08 ± 0.02
*t*	—	46.842	62.404	38.950
*P*value	—	<0.001	<0.001	<0.001

**Table 3:** Comparison of fetal growth and development ($\bar{x}$ ± *s*).

Groups	*n*	HC	BPD	FL	AC
Study group	98	31.65 ± 2.81	8.82 ± 0.76	6.79 ± 0.58	30.88 ± 3.29
Control group	100	32.94 ± 1.93	9.18 ± 0.53	7.02 ± 0.53	32.77 ± 2.38
*t*	—	3.772	3.873	2.914	4.638
*P*value	—	<0.001	<0.001	0.004	<0.001

**Table 4:** Comparison of ultrasound hemodynamic parameters ($\bar{x}$ ± *s*).

Index		Study group (*n* = 98)	Control group (*n* = 100)	*t*	*P*value
UA	RI	0.89 ± 0.18	0.66 ± 0.12	10.599	<0.001
	PI	1.21 ± 0.23	1.08 ± 0.13	4.909	<0.001

AoI	RI	0.71 ± 0.10	0.87 ± 0.17	8.051	<0.001
	PI	1.96 ± 0.25	2.32 ± 0.38	7.859	<0.001

DV	RI	0.63 ± 0.17	0.48 ± 0.12	7.184	<0.001
	PI	0.86 ± 0.19	0.64 ± 0.13	9.525	<0.001

PV	RI	0.68 ± 0.11	0.52 ± 0.08	11.722	<0.001
	PI	1.03 ± 0.18	0.83 ± 0.12	9.216	<0.001

**Table 5:** Comparison of fetal heart function parameters ($\bar{x}$ ± *s*).

Index		Study group (*n* = 98)	Control group (*n* = 100)	*t*	*P*
Ventricular IVCT	Left	48.33 ± 6.98	38.65 ± 5.18	11.097	<0.001
	Right	52.88 ± 12.08	42.61 ± 9.52	6.551	<0.001

Ventricular IVRT	Left	48.86 ± 7.02	40.91 ± 6.77	8.112	<0.001
	Right	49.98 ± 11.02	40.32 ± 8.13	7.029	<0.001

Ventricular MPI	Left	0.53 ± 0.11	0.42 ± 0.07	8.412	<0.001
	Right	0.57 ± 0.11	0.47 ± 0.09	7.007	<0.001

Valve *E*	Mitral	0.29 ± 0.05	0.34 ± 0.09	4.819	<0.001
	Tricuspid	0.32 ± 0.04	0.41 ± 0.11	7.621	<0.001

Valve *E*/*A*	Mitral	0.49 ± 0.14	0.58 ± 0.11	5.035	<0.001
	Tricuspid	0.51 ± 0.05	0.62 ± 0.14	7.333	<0.001

*Note.* Only parameters with statistically significant (*P* < 0.05) differences are shown. The values of left and right ventricular ET and mitral and tricuspid A values were not significant between the two groups (*P* > 0.05).

**Table 6:** Correlation of ultrasound parameters with clinical data.

Index	*r* value	*P*value
Systolic pressure		
UA PI	0.761	<0.01
UA RI	0.739	<0.01
AoI PI	−0.842	<0.01
AoI RI	−0.801	<0.01
DV PI	0.802	<0.01
DV RI	0.759	<0.01
PV PI	0.793	<0.01
PV RI	0.762	<0.01
Left ventricular IVCT	0.748	<0.01
Left ventricular IVRT	0.752	<0.01
Left ventricular MPI	0.838	<0.01
Right ventricular IVCT	0.747	<0.01
Right ventricular IVRT	0.749	<0.01
Right ventricular MPI	0.801	<0.01
Mitral valve *E*	−0.785	<0.01
Mitral valve *E*/*A*	−0.802	<0.01
Tricuspid valve *E*	−0.774	<0.01
Tricuspid valve *E*/*A*	−0.816	<0.01

*Note.* Only parameters with correlation (*P* < 0.05) are shown. There was no correlation between left and right ventricular ET and mitral and tricuspid A parameter values and systolic blood pressure (*P* > 0.05). All ultrasound parameters did not correlate with diastolic blood pressure and 24 h urine protein quantification (all *P* > 0.05).

**Table 7:** Comparison of umbilical artery blood flow parameters for different fetal growth and development ($\bar{x}$ ± *s*).

Groups	*n*	S/D	PI	RI
Study group A	39	3.89 ± 0.98	1.29 ± 0.33	0.79 ± 0.16
Study group B	59	2.50 ± 0.66	0.91 ± 0.31	0.63 ± 0.08
*t*	—	8.397	5.789	6.552
*P*value	—	＜0.001	＜0.001	＜0.001

*Note.* Study group A, fetal growth restriction; study group B, normal fetal growth.

**Table 8:** Comparison of fetal cardiac function parameters between the two groups ($\bar{x}$ ± *s*).

Items	Cut-off value	AUC	Sensitivity (%)	Specificity (%)	Youden index
S/D	3.53	0.883	63.88	96.85	0.607
PI	1.02	0.801	83.45	65.61	0.492
RI	0.71	0.842	75.02	86.42	0.616

*Note.* AUC refers to the area under the curve.

## Data Availability

The datasets used during the present study are available from the corresponding author upon reasonable request.
